The article "Arthroscopic Meniscal Repair: University Hospital Southampton Experience" was retracted in 2024. Reasons: no approval from an author; concerns about the authorship.

# Arthroscopic Meniscal Repair: University Hospital Southampton Experience

**DOI:** 10.7759/cureus.41813

**Published:** 2023-07-13

**Authors:** Nzubechukwu Ijezie, Hossam Fraig

**Affiliations:** 1 Surgery, Dorset County Hospital NHS Foundation Trust, Dorchester, GBR

**Keywords:** anterior, mensicus, fast-fix, arthroscopy knee, all-inside repair

## Abstract

Introduction

The meniscus plays an integral role in the proper functioning of the knee joint. Located between the articular surfaces of the tibia and femur, the meniscus functions to provide stability to the knee joint, even out axial load, absorb shock, and provide some lubrication to the knee joint. Accordingly, treatment of meniscal injuries aims to preserve as much meniscal tissue as possible to avoid the myriad complications that arise from its removal.

This study of the all-inside technique for meniscal repair evaluates the University Hospital Southampton experience by comparing our outcomes with the available literature.

Patients and methods

This is a retrospective study from January 2016 to December 2020. Records of patients were obtained through the preoperative assessment clinics network and electronic notes. The endpoints of the study were defined as patients who either were discharged, experienced failure of repair, i.e., symptomatic or magnetic resonance imaging (MRI) changes, or were offered re-surgery.

Results

Eighty-one patients, comprising 51 males and 30 females, were included in the study, and 85 repairs were performed. A steady increase in the number of procedures was observed year on year until the outbreak of COVID-19. The mean age of patients was 24.7 years, with a range of 39 years.

The medial meniscus was found to be injured more often than the lateral meniscus. The most commonly observed injury pattern was the bucket handle (BH) type. Anterior cruciate ligament (ACL) injury was found to be associated with meniscal injuries in around half of patients. The reason for this occurrence can be attributed to the ligamentous connection between the medial meniscus and the anterior cruciate ligament in the phenomenon described in the "unhappy triad."

On average, three FasT-Fix sutures were required per procedure.

Discussion and conclusion

After a follow-up of 11 months, 11 (13.6%) treated patients were noted to have failed repair, as defined by the endpoint criteria. Age and acuity were noted to not affect outcomes, and the results suggest that males are at higher risk of failed repair than females (p<0.05).

## Introduction

The meniscus, which is formed of cartilage, lies in the knee between the femur and tibia bones. By virtue of its location and properties, the gliding motion of these apparently opposing bones is seamless. Moreover, the composition of the meniscus lends itself to absorbing the shock from the weight transmitted through the knees from both above and below. Needless to say, the importance of the meniscus to the optimal functioning of the knee cannot be overstated. Consequently, the integrity of the meniscus is critical to ensuring seamless mobility and optimal functioning of the knee joint [1].

The article "Arthroscopic Meniscal Repair: University Hospital Southampton Experience" was retracted in 2024. Reasons: no approval from an author; concerns about the authorship.

To this end, various techniques have been trialed to conserve as much meniscal tissue as possible to prevent the many problems associated with mobility and stability of the knee joint that arise with the removal or injury to the meniscus. This is because there is evidence that degenerative alterations are directly proportional to the amount of meniscus removed [1], as several studies have demonstrated the advantages of repair over meniscectomy [2,3]. Following the evolution of methods, the FasT-Fix method has become one of the most accepted for treating meniscal tears. This method of repair, which utilizes the placement of mattress sutures through the meniscus, has been demonstrated to be safe and effective. The FasT-Fix technique was noted by one study to be safe and effective while providing very impressive results. In this study, Stryker's meniscal repair kit was the device used for repairs [4].

The aim of this study is to evaluate the University Hospitals Southampton experience and compare our outcomes with the available literature.

## Materials and methods

This is a retrospective study from January 2016 to December 2020. Records for the patients were obtained through the preoperative assessment clinics network and electronic notes.

Included in the study were all types of meniscal repairs (isolated or combined with anterior cruciate ligament repair (ACLR)) performed within the specified period, beyond which an endpoint was reached. The duration of follow-up after surgery was 11 months.

The endpoints of the study were defined as patients who either were discharged, experienced failure of repair, i.e., symptomatic or magnetic resonance imaging (MRI) changes, or were offered re-surgery. Surgical repair was performed by seven knee surgeons utilizing the FasT-Fix repair kit by Stryker. The collated data was analyzed using Statistical Package for the Social Sciences (SPSS) version 26 (IBM SPSS Statistics, Armonk, NY, USA), with a confidence interval of 95%.

Excluded from the study were patients with injuries to the knee joint devoid of meniscal involvement.

## Results

Of the 106 patients who presented to the hospital with meniscal and knee issues, 81 patients were included in the study. Eighty-five meniscal repairs were performed, with a rise in the number of repairs per year until the outbreak of the COVID-19 pandemic (Figure 1).

The article "Arthroscopic Meniscal Repair: University Hospital Southampton Experience" was retracted in 2024. Reasons: no approval from an author; concerns about the authorship.

**Figure 1:** Number of cases performed per year The curved line represents the actual number of cases performed. The straight line represents the projected number of cases. COVID-19: coronavirus disease 2019

In this study, there were 51 (63%) male patients and 30 (37%) female patients. The mean age of patients who were treated for meniscal injuries was 24.7 years, with a range of 39 years. Many of the patients who were treated for meniscal injuries were between 20 and 40 years old (Figure 2).

**Figure 2:** Patient demographics Age and gender distribution

Regarding the laterality of injuries, the medial meniscus was found to be injured in 60% of cases and the lateral meniscus in 35%, while about 5% had mixed injuries. There was a significant difference (p<0.05) in the occurrence of medial compared to lateral meniscal injuries. Meniscal injuries were approximately evenly distributed between the left and right sides at 52% and 48%, respectively (Figure 3).

**Figure 3:** Laterality and side of injury Left: laterality of injury, right: side of injury There was a significant difference in the occurrence of medial meniscal injuries compared to lateral (p<0.05) (Statistical Package for the Social Sciences (SPSS) version 26)

In terms of the type of meniscal injuries, half (n=42, 50%) were found to be bucket handle (BH). The other injury types identified were longitudinal tears, ramp, horizontal and radial tears, and hypermobility (Figure 4).

**Figure 4:** Injury type BH injury was the most commonly observed injury type, followed by longitudinal tears. BH: bucket handle

In addition to the injury patterns described above, anterior cruciate ligament (ACL) injury was found to be associated with 44 (54%) patients who were treated for injuries. Of these, 36 (82%) had reconstruction of the ACL in addition to meniscal repair (Figure 5).

**Figure 5:** ACL involvement Left: ACL injury, right: ACL reconstruction ACL: anterior cruciate ligament

On average, many patients required three FasT-Fix sutures to achieve satisfactory repair of their injury (Figure 6).

**Figure 6:** Number of FasT-Fix sutures per meniscal repair

After a follow-up of 11 months, 58 (71.6%) patients were discharged. Five patients were followed up, seven patients declined follow-up, and 11 patients were reported as "failed" as per the endpoint criteria.

## Discussion

After the 11-month follow-up, 11 patients were noted to have failed repair as per the endpoint criteria. Of these, one patient was excluded from the process, as they indicated not wanting to continue with further investigations or treatment. Of the 10 remaining patients, medial meniscal injuries comprised 70%. Overall, a failure rate of 13.6% was observed from the results of this retrospective study. The mean age in the failed repair cases was 35 years, with a range between 20 and 47 years. The majority of the patients who were reported as failed were male (n=7), with BH injury constituting 50% of failed injury patterns. Other patterns were longitudinal (n=3) and horizontal (n=2) tears. Of this cohort, 40% also had anterior cruciate reconstruction. Age and acuity were noted to not affect outcomes.

The article "Arthroscopic Meniscal Repair: University Hospital Southampton Experience" was retracted in 2024. Reasons: no approval from an author; concerns about the authorship.

Considerable variation between 70% and 94% in successful clinical outcomes for all-inside meniscal repair has been reported in the literature. For example, a success rate of 85% was reported in four studies [5-8], with other studies reporting failure rates from 9.5% to 17% after a follow-up of 18-30 months [9-11]. A meta-analysis of the literature for predictive prognostic factors such as age, patient sex, and time from injury to surgery found no significant effect on outcomes [12,13].

Although there is conflicting evidence on outcomes when concurrent anterior cruciate ligament reconstruction (ACLR) is performed, our data favored a better outcome when ACLR was also performed. There are different postulations on why this could be the case, with some asserting that it could be due to the vascularity associated with the ACL and the consequent inflammatory process that ensues from injury and repair. Another reason could be the added attention to detail of the surgeons performing these procedures.

Pujol et al. [14] reported a failure rate of 12.9% following meniscal repair with FasT-Fix after an average follow-up of 9.5 years, although the study did not find any effect of ACLR or laterality on the overall healing after meniscal repair was identified. After a follow-up of seven years, Bogunovic et al. [8] reported a failure rate of 16%, suggesting that a longer follow-up was required to elucidate survivorship after meniscal repair with FasT-Fix. Table 1 presents a comparison of studies on all-inside repair.

**Table 1:** Comparison of studies on all-inside repair

Authors	Year	Patients/studies	Failure rate	Duration of follow-up
Ardizzone et al. (systematic review)	2020	763/15	Overall: 29.3% (19% for devices still in use)	Average 13 months
Bogunovic et al.	2014	83	16%	>5 years
Costa et al. (systematic review and meta-analysis)	2021	38 articles	Pooled failure rate: 14.8%	-
Laurendon et al.	2017	87	13 (14.9%)	31 months
Majeed et al.	2015	136	23 (17%)	Average 9 months
Moses et al.	2017	51	12 (23.5%)	2 years
Nepple et al. (systematic review and meta-analysis)	2012	566/13	131 (23.1%)	>5 years
Nobile et al.	2020	54	10 (18.5%) within 1 year	4 years
Pujol et al.	2008	53	<12%	1 year
Turcotte et al.	2021	87	15 (17.2%)	2.7 years
Zimmerer et al.	2018	63	17 (27%)	12 years

Findings from Ardizzone et al. [15] posited that outcomes from all-inside repair for BH injuries might be less favorable compared to other techniques, perhaps based on the peculiarity of BH tears, as the zones of repair are not well reported in the literature. This could explain the frequency with which BH injuries present in "failed repair" patients.

The article "Arthroscopic Meniscal Repair: University Hospital Southampton Experience" was retracted in 2024. Reasons: no approval from an author; concerns about the authorship.

This study was limited by the sample size and the duration of follow-up. In addition, the heterogeneity of the sample population combined with variations in activity level and possible mechanisms of injury were not accounted for, even as recovery following rehabilitation would be expected to vary based on physiological status. Although negligible, variation between different surgeons could be assumed to have had an impact on outcomes and, therefore, is a limitation of this study. Furthermore, another limitation was the non-utilization of validated outcome scoring tools such as patient-reported outcome measures (PROMs) to limit the subjectivity of outcomes.

In comparison to other studies, there was no standardized endpoint, as each study had its own set of definitions for what constitutes an endpoint, which could skew the results.

## Conclusions

The failure rate after meniscal repair at 11 months with Stryker's meniscal repair kit is 13.6%. Age and acuity did not affect the overall outcome of the study, buttressing the finding that it is possible to preserve the meniscus across different age groups. While the medial meniscus was significantly more injured than the lateral meniscus, there was no difference in what side the knee injury occurred.

There was an increase in the number of cases performed year on year until the outbreak of the COVID-19 pandemic and the shutdown of services in 2020. Of all injury types identified, BH injury was the most prevalent. Furthermore, ACL injuries, which often required reconstruction, were associated with these injuries and linked to better repair outcomes. On average, three sutures were required for the repair of injuries regardless of laterality.
